The article "Association between obesity and abnormal Papanicolau(Pap) smear cytology results in a resource-poor Nigerian setting" was published in 2020. Journal: BMC Womens Health.

# Association between obesity and abnormal Papanicolau(Pap) smear cytology results in a resource-poor Nigerian setting

**DOI:** 10.1186/s12905-020-00984-w

**Published:** 2020-06-09

**Authors:** Silas Onyemaechi Okoro, Leonard Ogbonna Ajah, Peter Onubiwe Nkwo, Uzochukwu U. Aniebue, Benjamin Chukwuma Ozumba, Chibuike Ogwuegbu Chigbu

**Affiliations:** Department of Obstetrics and Gynaecology, Faculty of Medical Sciences, University of Nigeria, Ituku-Ozalla Campus, Enugu, Nigeria

**Keywords:** Obesity, Pap smear cytology, Cervical epithelial cell abnormalities, South-East Nigeria

## Abstract

**Background:**

Though obesity is associated with some malignancies, its association with cervical cancer is still inconclusive. This study was aimed at determining if there was an association between obesity and cervical epithelial cell abnormalities (CEA).

**Methods:**

This was a cross-sectional comparative study of obese and non-obese women at the Cervical Cancer Screening Clinic, University of Nigeria Teaching Hospital (UNTH), Enugu between January, 2012 and June, 2013. The participants whose body mass index (BMI) were ≥ 30 kg/m^2^ were classified as obese (200 women) while those whose BMI were < 30 kg/m^2^ were classified as non-obese (200 women) and the two groups were consecutively recruited at the ratio of 1:1. Pap smear cytology, random blood sugar (RBS) and human immune-deficiency virus (HIV) screening was done for all the participants. Data was analyzed with SPSS version 20. Categorical variables were analyzed using McNemar’s test and Chi-squared test. Logistic regression analysis was used to determine the influence of socio-demographic characteristics on cervical epithelial cell abnormalities. The level of significance was set at ≤0.05.

**Results:**

Among the obese women, 152(76%) had negative for intra-epithelial lesion or malignancy (NILM) while 48(24%) had cervical epithelial cell abnormalities (CEA). Also 182(91%) non-obese women had NILM while the remaining 18(9%) had CEA. The prevalence of CEA among all the study participants was 16.5%. There was an association between obesity and CEA[OR (95%CI) = 1.353(1.013–1.812); *P*-value = 0.04].CEA were significantly more common among women who were 40 years and above and single/separated women as well as widows (*P*-value = < 0.05).

**Conclusion:**

There was an association between obesity and CEA. This underscores the need for a positive behavioural change among women in order to stem the tide of this public health problem.

## Background

There is currently an increase in the prevalence of obesity globally. The World Health Organization (WHO) estimates that more than 1 billion people are overweight, with 300 million people meeting the criteria for obesity [1].Obesity is defined as body mass index of more than 30 kg/m^2^ [1]. Obesity is regarded as a risk factor for many cancers [2, 3]. The relationship between obesity and hormonal levels stimulates interest because of its role in hormone dependent cancers [4]. Previous studies have shown that obesity may increase the risk of cervical cancer [5–8]. Cervical adenocarcinoma has been linked to hormonal risk factors and has been reported to be increasing in incidence in recent years [4, 9, 10]. A recent meta-analysis showed a weak association between obesity and cervical cancer [11]. However the authors of this meta-analysis requested for more studies in this topic in order to strengthen or refute the current evidence.

The article "Association between obesity and abnormal Papanicolau(Pap) smear cytology results in a resource-poor Nigerian setting" was published in 2020. Journal: BMC Womens Health.

Obesity has also been shown to not only increase the incidence but mortality due to cervical cancer [7, 12]. This may be attributed to lack of or late cervical cancer screening, co-morbid illnesses, or poor response to treatment by obese women [12, 13]. Recent evidence indicates that a weight loss of more than 9 kg in women is associated with a quarter reduction in all causes of mortality such as diabetes, cardiovascular disorders and cancer [14]. Cervical cancer is a major public health threat to women in many resource-poor countries including those in sub-Saharan Africa. In Nigeria, the crude incidence and age-standardized incidence of cervical cancer are 17.1/100,000 and 29.0/100,000 women respectively [15]. Current estimates indicate that annually, 14,089 women are diagnosed with cervical cancer and 8240 die from the disease [15]. This is very high and measures to stem the tide of high cervical cancer burden in Nigeria, need urgent implementation. It is therefore imperative to recognize not only the dependent causal role of human papilloma virus (HPV) in cervical cancer but the co-factors. Such co-factors are the exposures and risk factors that, when present with HPV infection, potentiates the development of cervical cancer [16].

Despite the high incidence of cervical cancer in Nigeria, the awareness and uptake of cervical cancer and its screening is very low [17, 18]. Papanicolaou(Pap) smear testing is a common cervical cancer screening method in Nigeria [19]. It is a secondary preventive method which is used globally in the diagnosis of pre-malignant and malignant lesions of the cervix [20]. Pap smear cytology screening facilities are available in both urban and rural areas in Nigeria. Though Pap smear cytology is associated with errors, a previous report in South-East Nigeria showed an overall accuracy of Pap smear cytology screening at between 90 and 97% [20, 21]. Therefore Pap smear cytology screening will be useful for population studies in this subject matter in Nigeria. Based on medline search, no previous study evaluated the association between obesity and cervical epithelial cell abnormalities in Nigeria. It is because of these reasons that this study was embarked upon. This study was aimed at determining if there was an association between obesity and cervical epithelial cell abnormalities among the women who presented for Pap smear cytology in Enugu, South- East Nigeria.

The article "Association between obesity and abnormal Papanicolau(Pap) smear cytology results in a resource-poor Nigerian setting" was published in 2020. Journal: BMC Womens Health.

## Methods

### Study area

Enugu State has Enugu as its capital. It is one of the five states that make South-East Nigeria. Enugu state is predominantly inhabited by Igbo communities. It has the population of 3,267,837 people according to 2006 population census [22]. The University of Nigeria Teaching Hospital (UNTH) is a federal tertiary health institutions that is sited at Ituku-Ozalla. This hospital is about 21 km from Enugu metropolis. UNTH serves the people of South-East, South-South and northern states. Highly specialized cases are occasionally referred from Cameroun. The hospital has a cancer screening center. The cervical cancer screening clinic gets referrals from the gynaecology clinic and other clinics in UNTH and from peripheral hospitals.

### Study design

This study was a cross-sectional comparative type that was conducted at UNTH between January, 2012 and June, 2013.The obese and non-obese women were purposively recruited at the Gynaecology clinic, UNTH. The height of each patient was usually checked at the first visit of every patient at the clinic. But the weight of patients were routinely checked at every visit. It was from each patient’s record that her weight and height were collated and Body Mass Index (BMI) was calculated. Also data on age, parity, residential address and educational qualification was collated from the patients. The women who met the eligibility criteria were encouraged to go to the cervical cancer screening clinic for counseling and screening of the consenting participants. At the cervical cancer screening clinic, the women were counselled on cancer of the cervix, the screening procedures, and objectives of the study, following which, consent to participate in the study was sought and obtained. Data on number of life sexual partners and history of smoking was collated from the consenting study participants. For the purpose of this study, a woman was said to be obese if her BMI was ≥30 kg/m^2^ while she was said to be non-obese if her BMI was < 30 kg/m^2^. Pap smear cytology, random blood sugar (RBS) and human immune-deficiency virus (HIV) screening were also done on all the participants. Standard precautions [23], were taken prior to sample collection from the participants. The ecto-cervical and endo-cervical samples were collected with Ayre spatula and cytobrushes respectively. A double-slide technique in which the ecto-cervical and endo-cervical samples were placed separately on each slide was performed. The Pap smear cytology result was reported using the Bethesda 2001 system [24]. For the purpose of this study, the Pap smear cytology result was negative when it was negative for intra-epithelial lesion or malignancy but positive when there was cervical epithelial cell abnormality. Also for the purpose of this study, the women with RBS of > 125 mg/dl were classified as being abnormal while those with RBS ≤125 mg/dl were classified as being normal. The eligible participants were consecutively recruited and classified into two groups in the ratio of 1:1. Group 1 participants were those whose BMI were ≥ 30 kg/m^2^ (obese women) while the group 2 participants were those whose BMI was < 30 kg/m^2^(non-obese women).The two groups of participants were matched for age, parity, residential address, educational qualification and number of life sexual partners. Also for the purpose of this study, number of life sexual partners means the total number of sexual partners the study participants had from their first sexual intercourse to the time this study was conducted. The ages of the two groups of participants were matched at interval of 21–30 years, 31–40 years, 41–50 years, 51–60 years and 61–70 years. The educational qualification of the participants were also matched for no formal education, primary education, secondary education and tertiary education respectively. The parity distribution of the women were matched as nulliparity, primiparity, multiparity and grandmultiparity. The residential addresses of the respondents were matched for rural and urban respectively. The number life sexual partners were matched as 1, 2, 3 and ≥ 4. A pro forma was used to collate information on the socio-demographic characteristics and the screening results of the participants. Exclusion criteria comprised women who were less than 21 years, pregnant women, women who had abnormal blood sugar results, HIV positive women, smokers and those within 6 weeks post-partum as well as the women who, despite adequate counselling, declined to participate in the study. The primary outcome measure was the proportion of obese and non-obese women who had cervical epithelial cell abnormalities. The secondary outcome measures were the effect of socio-demographic characteristics on cervical epithelial cell abnormalities development.

The article "Association between obesity and abnormal Papanicolau(Pap) smear cytology results in a resource-poor Nigerian setting" was published in 2020. Journal: BMC Womens Health.

The sample size (n) was determined using the formula for cross-sectional comparative studies [25]:

$$ \mathrm{n}=\frac{\mathrm{r}+1}{\mathrm{r}}.\frac{\ \left(\mathrm{P}\ast \right)\left(1\hbox{-} \mathrm{P}\ast \right){\left({\mathrm{Z}}_{\upbeta}+{\mathrm{Z}}_{\upalpha /2}\right)}^2}{{\left({\mathrm{P}}_1\hbox{-} {\mathrm{P}}_2\right)}^2} $$

Where: n = sample size; r = ratio of cases to control=1; P* = Average proportion of exposed cases = $\frac{\mathrm{Proportion}\ \mathrm{of}\ \mathrm{exposed}\ \mathrm{cases}+\mathrm{proportion}\ \mathrm{of}\ \mathrm{control}\ \mathrm{exposed}}{2}$;

P* = 0.625 [26]

Z_β_ = Standard normal variate for power of 80% = 0.84; Z_α/2_ = Standard normal variate for level of significance and at 95% confidence interval, Z_α/2_ = 1.96; P_1_ = Proportion of cervical epithelial cell abnormalities among overweight and obese women =0.67 [26]; P_2_ = Proportion of CEA among underweight women = 0.27 [26]

Adding 10% attrition rate, the sample size for each of the groups was 141.

Data was analyzed with Statistical Package for Social Sciences version 20 software (IBM SPSS Inc., Chicago, IL, USA). Categorical variables were analysed using McNemar’s test and Chi-squared test. Logistic regression analysis was used to determine the influence of socio-demographic characteristics on cervical epithelial cell abnormalities. The level of significance was set at ≤0.05. The ethical clearance for this study was obtained from the Health Research Ethics Committee of UNTH.

## Results

A total of 7583 patients were seen at the gynaecology clinic within the study period. Six hundred and five patients were purposively picked and encouraged to come to the cervical cancer screening clinic for this study. However, it was only 509 patients that actually came to the cervical cancer screening clinic from the gynaecology clinic and were counseled for the study. A total of 659 women, who accounted for 58% of clients that had Pap smear cytology at the cervical cancer screening clinic within the study period, were referred from other clinics and so were not involved in this study. Furthermore, 78 women, who accounted for 6.9% of clients that had Pap smear cytology within the study period, were part of those that were invited from the gynaecology clinic but did not meet the inclusion criteria for this study. Figure 1 shows the distribution of 509 women who were counseled for this study. A total of 200 obese women and 200 non-obese women were recruited for the study. So the results of these 400 participants were analysed. However 109 women were excluded from the study due to non-consent, smoking, abnormal blood sugar levels and HIV infection. Table 1 shows comparison of the socio-demographic characteristics between the obese and non-obese women. There was no statistical significant difference between the obese and non-obese women on the socio-demographic characteristics. Table 2 shows the Pap smear cytology results of the obese and non-obese women. A total of 152(76%) obese women had negative for intra-epithelial lesion or malignancy (NILM) while 48(24%) had CEA. However, a total of 182(91%) non-obese women had NILM, but 18(9%) had CEA. The prevalence of cervical epithelial cell abnormalities among all the study participants was 16.5%. Table 3 shows the association between obesity and cervical epithelial cell abnormalities. There was an association between obesity and cervical epithelial cell abnormalities in this study [OR (95%CI)1.353(1.013–1.812); *P*-value = 0.04]. The effect of socio-demographic characteristics of the participants on cervical epithelial cell abnormalities is shown on Table 4. Cervical epithelial cell abnormalities were significantly more common among women who were 40 years and above, women who had multiple sexual partners, single/separated women and widows. Table 5 shows the logistic regression of the influence of socio-demographic characteristics on cervical epithelial cell abnormalities. Age, marital status and occupation had a significant influence on cervical epithelial cell abnormalities.

The article "Association between obesity and abnormal Papanicolau(Pap) smear cytology results in a resource-poor Nigerian setting" was published in 2020. Journal: BMC Womens Health.

**Fig. 1:** Flow chart of how the obese and non-obese women were recruited

**Table 1:** Comparison of the socio-demographic characteristics between the obese and non-obese women

Socio-demographic characteristics	Obese women ***N*** = 200	Non-obese women ***N*** = 200	OR (95% CI)	***P***-value
**Age(years)**			1.00 (0.75–1.33)	0.94
21–30	32	32		
31–40	68	68		
41–50	54	54		
51–60	37	37		
61–70	9	9		
**Marital status**			1.05 (0.79–1.40)	0.78
Married	180	170		
Single	6	10		
Separated	8	13		
Widow	6	7		
**Residential address**			0.87 (0.65–1.16)	0.36
Rural	55	71		
Urban	145	129		
**Educational qualification**			0.96 (0.72–1.28)	0.83
No formal	14	24		
Primary	38	32		
Secondary	93	101		
Tertiary	55	43		
**Number of life sexual partners**			0.92 (0.69–1.23)	0.62
1	46	54		
2	97	83		
3	38	45		
≥ 4	19	18		
**Parity**			1.06 (0.80–1.42)	0.72
0–1	41	35		
2–4	71	87		
≥ 5	88	78		
**Occupation**			1.11 (0.83–1.48)	0.52
Unemployed	38	28		
Farming	50	67		
Trading	17	17		
Civil service	19	26		
Teaching	36	26		
Artisans	16	18		
Professionals	24	18		

*OR* Odds ratio, *CI* Confidence Interval

**Table 2:** The Pap smear cytology results of the obese and non-obese women

Pap smear cytology	Obese women [***N*** = 200(%)]	Non-obese women [***N*** = 200(%)]
NILM	152 (76)	182 (91)
ASCUS	10 (5)	6 (3)
LSIL	25 (12.5)	7 (3.5)
HSIL	13 (6.5)	5 (2.5)
**Prevalence of cervical epithelial cell abnormalities among the study participants was 16.5%**		

*NILM* Negative to squamous intraepithelial lesion or malignancy, *ASCUS* Atypical squamous cells of undetermined significance, *LSIL* Low-grade squamous intraepithelial lesion, *HSIL* High-grade squamous intraepithelial lesion

The article "Association between obesity and abnormal Papanicolau(Pap) smear cytology results in a resource-poor Nigerian setting" was published in 2020. Journal: BMC Womens Health.

**Table 3:** Association between obesity and cervical epithelial cell abnormalities

Pap smear cytology	Obese women *N* = 200(%)	Non-obese women *N* = 200(%)	OR (95%CI)	*P*-value
Positive	48 (24)	18 (9)	1.353 (1.013–1.812)	**0.04**
Negative	152 (76)	182 (91)		

*OR* Odds ratio, *CI* Confidence Interval

**Table 4:** The effect of socio-demographic characteristics of the participants on cervical epithelial cell abnormalities

Socio-demographic characteristics	Cervical epithelial cell abnormalities		X^**2**^	***P***-value
	Negative [***N*** = 334(%)]	Positive [***N*** = 66(%)]		
**Age (years)**			9.291	**0.002**
≤ 40	184 (55.1)	16 (24.2)		
≥ 41	150 (44.9)	50 (75.8)		
**Marital status**				**0.001**
Married	312((93.4)	48 (72.7)	10.901	
Single/separated/widow	22 (6.6)	18 (27.3)		
**Residential address**			1.740	0.187
Rural	105 (31.4)	31 (47)		
Urban	229 (68.6)	35 (53)		
**Educational qualification**			0.001	0.969
≤ Primary	89 (26.6)	19 (28.8)		
≥ Secondary	245 (73.4)	47 (71.2)		
**Number of life sexual partners**			4.124	**0.042**
1	93 (27.8)	7 (10.6)		
≥ 2	241 (72.2)	59 (89.4)		
**Parity**			0.044	0.834
≤ 1	66 (19.8)	12 (18.2)		
> 1	268 (80.2)	58 (81.8)		
**Occupation**			4.331	**0.037**
Unemployed	47 (14.1)	19 (28.8)		
Working group	287 (85.9)	47 (71.2)

**Table 5:** Logistic regression of the influence of socio-demographic characteristics on cervical epithelial abnormalities

Socio-demographic characteristics	Influence on cervical epithelial cell abnormalities		
	Coefficient	Standard Error	***P***-value
Age	2.164	0.045	0.0001
Marital status	2.085	0.063	0.001
Occupation	1.120	0.147	0.045
Constant	0.728	0.087	
Cox and Snell R square	0.039	0.513	

## Discussion

This study showed that the prevalence of cervical epithelial cell abnormalities among the study participants was 16.5%. It also showed that there was an association between obesity and cervical epithelial cell abnormalities. Cervical epithelial cell abnormalities were significantly more common among women who were 40 years and above, single/separated women and widows (*P*-value = < 0.05).

The 16.5% prevalence of cervical epithelial cell abnormalities recorded in this study is essentially similar to 11.2 and 11.3% previously reported in Abakaliki, South-East Nigeria and Sokoto, Northern Nigeria respectively [17, 27]. It is however less than 29.3 and 34.6% previously reported in Nnewi, South-East Nigeria and Ife, South-West Nigeria [28, 29]. The high prevalence of cervical epithelial cell abnormalities in Nigeria could be attributed to very poor uptake of human papilloma virus (HPV) vaccine by the target population, early sexual exposure and involvement of multiple sexual partners by many women in resource-poor countries [30]. The association between obesity and cervical epithelial cell abnormalities in this study is supported by meta-analysis by Poorolajal and Jenabi which showed a weak relationship between obesity and cervical neoplasia [11]. It is also supported by a study by Lee et al., in South Korea which showed a positive association between cervical cancer and increasing body mass index and sedentary life style [26]. Although HPV is an established cause of cervical neoplasia [31], the recent evidence has shown that the cause of cervical neoplasia is multi-factorial [32]. Even though the real mechanism of obesity in increasing the cervical cancer risk is not known, the possible mechanisms comprise inflammation-associated carcinogenesis and increased levels of endogenous hormones [33]. These endogenous hormones include sex steroids, insulin and insulin-like growth factor [34]. Cervical epithelial cell abnormalities being significantly more common among older women in this study is supported by previous reports in Ife, South-West Nigeria and South Korea [30, 31]. This could be due to higher risk of coital exposure and longer exposure to human papilloma virus infection among the older women when compared with younger women. More so, the significant proportion of unemployed women having cervical epithelial cell abnormalities in this study could be due to these group of women being prone to risky sexual behaviours like early sexual exposure, unprotected intercourse and involvement of multiple sexual partners.

The article "Association between obesity and abnormal Papanicolau(Pap) smear cytology results in a resource-poor Nigerian setting" was published in 2020. Journal: BMC Womens Health.

Cervical epithelial cell abnormalities being more common among single and separated women as well as widows when compared with married women in this study can be adduced to single/ separated women and widows being prone to multiple sexual partners when compared with married women. However, the poor association between the cervical epithelial cell abnormalities and women who had multiple sexual partners in this study is contrary to the study by Getnet et al., in Ethiopia [35]. Parity not having significant effect on cervical epithelial cell abnormalities in this study is contrary to previous reports [35, 36]. This could be due to small sample of nulliparous and primiparous women among the participants in this study.

This study was strengthened by the recruitment of women who were non-diabetics, non-smokers and who did not have HIV infection. However the absence of randomization in the selection of the study participants in this study may have introduced bias thereby weakening the study. Even though the accuracy of Pap smear cytology is high in this environment [21, 37], there can still be errors thereby weakening the validity of the results. Therefore HPV testing, colposcopy and biopsy would have increased the degree of accuracy of the results. Some aspects of information sought from the study participants were also prone to recall bias. This was a hospital-based study in which its findings may not be a true reflection in the larger community.

## Conclusion

There was an association between obesity and cervical epithelial cell abnormalities. Cervical epithelial cell abnormalities were significantly more common among women older than 40 years, single/ separated women and widows and unemployed women. This underscores the need for a positive behavioural change among women in order to stem the tide of this public health problem. Population based studies are expected in this subject matter to further strengthen or refute the findings from this study.

## Data Availability

The data and materials for this publication are in possession of the the lead author, Dr. Silas Onyemaechi Okoro and he can be contacted through his e-mail: okoroonyemaechi@yahoo.com.

## Abbreviations

ASCUS: Atypical squamous cells of undetermined significance
CEA: Cervical epithelial cell abnormalities
CI: Confidence Interval
HIV: Human Immune deficiency virus
HPV: Human papilloma virus
HSIL: High-grade squamous intraepithelial lesion
LSIL: Low-grade squamous intraepithelial lesion
NILM: Negative to squamous intraepithelial lesion or malignancy
OR: Odds ratio
SPSS: Statistical Package for Social Sciences
UNTH: University of Nigeria Teaching Hospital, Ituku-Ozalla Enugu
